# Perceptions of health professionals regarding minimally invasive tissue sampling (MITS) to identify the cause of death in stillbirths and neonates: results from a qualitative study

**DOI:** 10.1186/s40748-019-0112-x

**Published:** 2019-10-25

**Authors:** Anam Feroz, Anum Shiraz Ali, Mohsina Noor Ibrahim, Elizabeth M. McClure, Shiyam Sunder Tikmani, Sayyeda Reza, Zahid Abbasi, Jamal Raza, Haleema Yasmin, Khadija Bano, Afia Zafar, Sameen Siddiqi, Robert L. Goldenberg, Sarah Saleem

**Affiliations:** 1 Department of Community Health Sciences, The Aga Khan University, Stadium Road, PO Box 3500, Karachi, 74800 Pakistan; 2 National Institute of Child Health, Karachi, Pakistan; 3 RTI International, Durham, USA; 4 Department of Obstetrics and Gynecology, Jinnah Post-graduate Medical Center, Karachi, Pakistan; 5 Department of Pathology & Laboratory Medicine, The Aga Khan University, Stadium Road, PO Box 3500, Karachi, 74800 Pakistan; 6 Department of Obstetrics and Gynecology, Columbia University, New York, USA

**Keywords:** Minimal invasive tissue sampling, Cause of death, Neonates, Stillbirth, Health professionals, Acceptability, Qualitative study

## Abstract

**Background:**

Pakistan is considered to be one of the riskiest places in the world for childbirth as measured by its high stillbirth and neonatal mortality rates. Complete diagnostic autopsy remains the gold standard to determine the cause of death (CoD); however, it is not routinely implemented due to religious objections, sociocultural beliefs, limited resources and low demand from physicians and families. Recently, minimally invasive tissue sampling (MITS) using needle biopsies of multiple tissues to obtain tissue for histological examination and organism identification with PCR has been developed and promoted to determine CoD in low-resource areas. To ensure successful implementation of MITS, it is important to understand health professionals’ attitudes and perceptions related to MITS.

**Methods:**

A qualitative study was conducted at the National Institute of Child Health (NICH), Karachi, Pakistan. Focus group discussions (FGDs) and Key-informant interviews (KIIs) were conducted with health professionals including doctors, nurses, trainees, clinicians, bioethics experts and public health experts to explore their perceptions and views on acceptability of MITS. Data were analyzed using NVivo 10 software.

**Results:**

A total of 12 interviews (FGDs = 4; KIIs = 8) were conducted. Four overarching themes were identified: (I) acceptability of MITS; (II) perceived benefits of the MITS procedure; (III) factors facilitating the implementation of MITS; and (IV) health system requirements for implementing the MITS procedure. Generally, MITS was considered as a positive development for the health system. Diagnostic accuracy and identification of less common causes of death were highlighted as two main benefits of the MITS procedure. The study highlighted a number of facilitators for the acceptability of MITS including effective counseling, building trust with parents, fast procedure time, and approaching families within a few hours of death. In addition, lack of skilled staff, poorly equipped healthcare facilities and the potential high cost to conduct MITS were identified as challenges for the implementation of MITS.

**Conclusions:**

This formative research provided a unique opportunity to explore health professionals’ views and attitudes towards the MITS procedure. Such insights are crucial to ensure successful implementation and integration of a new technique into the existing health system. The research identified the factors influencing the acceptability of MITS among health professionals in Pakistan. The study also informed factors that could help facilitate the implementation of the MITS procedures in the context of Pakistan and similar settings.

## Plain English language summary

The high numbers of stillbirths and neonatal deaths remains a neglected health issue in Pakistan as well as in a number of other low- and-middle-income countries. Complete diagnostic autopsy (CDA), a gold standard methodology, improves our understanding of the disease processes related to neonatal death and stillbirth. Recently, a minimally invasive tissue sampling (MITS) technique has been developed and promoted to determine CoD in low-resource areas. To ensure successful implementation of MITS, it is important to understand health professionals’ attitudes and perceptions related to MITS. A qualitative study was conducted at the National Institute of Child Health (NICH), Karachi, Pakistan, using focus group discussions and key informant interviews with health professionals to explore their perceptions and views on the acceptability of MITS. Generally, MITS was considered as a positive development for the health system. The research identified the factors influencing and facilitating the acceptability of MITS among health professionals in Pakistan.

## Background

According to global health statistics, approximately 2.6 million neonatal deaths occur every year and the number of stillbirths is similar. Approximately 75% of stillbirths and neonatal deaths occur in sub-Saharan Africa and south Asia [1, 2]. In 2018, Pakistan has been considered one of the riskiest places in the world for childbirth (2), as measured by its high stillbirth rate (43/1000 births) and neonatal mortality rate (46/1000 livebirths) [1]. Risk factors for stillbirths include lack of access to appropriate antenatal and obstetric care, poor maternal health, and low socioeconomic status [3, 4]. The leading causes of neonatal mortality include preterm birth complications (36%), intrapartum related events (22%), sepsis (18%), congenital abnormalities (6%), and pneumonia (6%) [5]. For both neonatal deaths and stillbirths, specific infections and conditions which cause these deaths are often not identified and have largely been under-reported [6]. The high numbers of stillbirths and neonatal deaths remains a neglected health issue in Pakistan as well as in a number of other low- and middle-income countries (LMICs). To meet the United Nations’ Sustainable Development Goals of good health and well-being and ending preventable newborn and child deaths, it is crucial to identify the causes of deaths (CoD) in stillbirths and neonates [7].

Complete diagnostic autopsy (CDA), a gold standard methodology, improves our understanding of the disease processes related to neonatal death and stillbirth [8]. However, in LMICs such as Pakistan, full autopsies on neonates and stillbirths are rarely conducted to identify a definitive CoD due to cultural, financial, religious, and physical barriers [9, 10]. As a result, the majority of the families and health professionals with a perinatal death are left without understanding the CoD. Minimally invasive tissue sampling (MITS) is being explored as an alternate method to CDA to investigate the cause of stillbirth and neonatal death [11, 12]. MITS involves body inspection and recording of basic anthropometric data, body palpation, body imaging and a series of post-mortem needle punctures using biopsy needles to obtain body fluids and tissue samples of lungs, brain, liver and other organs, within the first few hours after death. The samples are then sent to laboratories for a thorough histopathological and microbiological examination that would help identify the CoD [11, 13]. In Mozambique, the validation of MITS compared to CDA has been conducted and the results showed a moderate to substantial concordance between the two methods (Kappa values ranging from 0.40 to 0.78) [13, 14]. Therefore, MITS is being investigated as a suitable alternative for CDA, especially in regions where the latter may not be acceptable or feasible [10].

Health professionals often have close interactions with families of deceased fetuses and infants around the time of death for several purposes such as informing them about their child’s health status, and counseling and taking consent for various diagnostic procedures [13]. Therefore, when introducing a new procedure such as MITS, it is important to understand health professionals’ perceptions and attitudes related to MITS (including the consent process) in order to ensure successful integration of this new technique into the existing health system.

We undertook a qualitative research study to explore health professionals’ attitudes towards MITS, the perceived benefits of MITS, and the key facilitators and health systems’ requirements for the implementation of MITS in the context of Pakistan. This study was conducted in preparation for a larger study, the “Project to Understand and Research Preterm Pregnancy Outcome in South Asia (PURPOSe)” [6]. The study findings obtained in this formative research will inform the development of feasible approaches to improve the consent processes and implementation of the MITS procedure. The study protocol [11] and the perceptions of parents and religious leaders about MITS are published elsewhere [15].

## Methods

### Study design and setting

This formative research employed an exploratory qualitative research design using semi-structured interviews and a purposive sampling approach. The details are described in the published study protocol [11]. The study was conducted at the National Institute of Child Health (NICH), Karachi, Pakistan, because of their well-established pediatric care protocols and willingness to participate in the study.

Focus group discussions (FGDs) with healthcare professionals were conducted at the meeting room of the NICH hospital, while key-informant interviews (KIIs) were conducted at the respective locations of the key-informants. The aim of the FGDs and KIIs was to explore and understand the acceptability of the MITS conducted in one procedure among healthcare professionals, public health experts, clinicians, and bioethics experts.

### Study participants

Healthcare providers working at the NICH hospital were purposively sampled for FGDs. All types of healthcare providers including residents, consultants, staff nurses and trainees were represented. FGDs with healthcare providers were of the meeting rooms at NICH. A trained moderator facilitated the focus groups.

Public health experts, clinicians, and bioethics experts were purposively sampled for KIIs. We emailed letters of invitation to KIs for the qualitative study. A few KIIs were arranged at NICH and others took place at locations preferred by the interviewees.

### Interview guide

A semi-structured interview guide was developed to explore healthcare professionals’ views and attitudes towards MITS, with a focus on the acceptability of MITS among healthcare professionals, perceived benefits, barriers to and factors facilitating the implementation and health systems requirements for implementing MITS. The detailed interview guide that was used to conduct this study is provided (Appendix). Before beginning the interview, the qualitative researchers first described the autopsy and the MITS procedures (Table 1).

**Table 1:** Overview of open autopsy and MITS procedure

Full autopsy	
- Body inspection and recording of basic anthropometric data; body weight, height/length, mid-upper arm circumference, head circumference, lower leg length and foot length	
- Extensive examination of internal organs begins with the creation of a Y or U- shaped incision from both shoulders joining over the sternum and continuing down to the pubic bone	
MITS	
- Body inspection and recording of basic anthropometric data; body weight, height/length, mid-upper arm circumference, head circumference, lower leg length and foot length	
- Body palpation by a MITS specialist.	
- Imaging/photography by a MITS technician	
- Biopsy needles to obtain samples of lung, brain, liver and other organs for histopathologic and microbiologic examination to help determine COD	

### Data collection

A free flow of information was encouraged, using probes from these discussions to obtain healthcare professionals’ perceptions of the MITS procedure. Interviews were conducted face-to-face in Urdu (FGDs = 4) or English (KII = 8) according to the participants’ preference and were audio recorded following consent from study participants. Interviews were conducted by two experienced qualitative researchers (AF & SR), who are part of the investigating team. Detailed field notes were also taken during each interview to capture non-verbal language and cues. KIIs lasted between 20 and 40 min; FGDs lasted 30 min to 1 h and consisted of 8 participants per group.

### Analysis

Study data were analyzed using thematic analysis facilitated by NVivo version 10 (QSR International, Pty Ltd) software. Data were collected and analyzed through an iterative process and data collection was ceased once saturation was achieved. First, all the audio recordings were translated and transcribed from the local language (Urdu) into English, and then the transcriptions were uploaded in the software. Transcripts were read several times to develop an interpretation of the participants’ perceptions towards MITS. Focus groups and KIIs were coded as one data set. Two investigators coded a subset of transcripts independently using separate NVivo files that were then combined to match codes, and agreement was sought on a coding framework. The remaining transcripts were then independently coded according to the framework. Codes were formulated inductively from the transcripts. Coding discrepancies were discussed and resolved to reduce researchers’ biases. Codes were then analyzed under major themes. The interview guide was used to outline major themes. Final overarching themes were discussed and reviewed by both investigators. To ensure the credibility of the research, study data were triangulated by the data sources (health care providers, public health experts, clinicians, bioethics experts) and data collection methods (FGDs and KIIs), to compare alternative perspectives and to assess any inconsistencies.

### Ethical considerations

Ethical approval for this study was obtained from the NICH hospital [11/2018] and Aga Khan University Ethical Review Committee (AKU-ERC) – [5358-CHS-ERC- 18]. Before the interview, informed consent was obtained from informants and focus group participants in which they agreed that the interview could be audio-recorded and written notes could be taken to record interviewee expressions and statements. Participants were assured that their anonymity would be maintained and no identifying features would be mentioned on the transcript.

## Results

A total of 12 semi-structured interviews were conducted between July 2018 and August 2018. Four FGDs were conducted with healthcare professionals working at NICH, with eight participants in each FGD. Eight KIIs were conducted with public health experts (*n* = 2), bioethics experts (n = 2) and clinicians (*n* = 4) (Table 2). All the participants (*n* = 40) who were approached by the study team agreed to participate.

**Table 2:** Study Participants

Focus Group Discussions with Healthcare Providers	Total FGDs =4; *n* = 32
Senior Health Care Providers (RMOs, Senior Consultants, Head Nurses)	2 groups (8 participants in each group)
Junior Health Care Providers (MCPS & FCPS Trainees, Staff Nurses)	2 groups (8 participants in each group)
Key Informant Interviews with Clinicians	Total KIIs = 4; n = 4
Gynecologists	2 KIIs
Neonatologists	2 KIIs
Key Informant Interviews with Bioethics Experts	Total KII = 2; n = 2
Expert from Clinical Trials Unit	1 KII
Behavioral and Social Science Expert	1 KII
Key Informant Interviews with Public Health Experts	Total KII = 2; n = 2
Population Health Expert	1 KII
Community Health Expert	1 KII

Based on the data collection and thematic analyses, four overarching themes were identified: (I) acceptability of MITS among health professionals; (II) perceived benefits of MITS procedure; (III) factors facilitating the implementation of MITS; and (IV) health system requirements for implementing MITS. These themes are presented in Table 3.

**Table 3:** Themes and sub-themes

Theme	Sub-theme
Acceptability of MITS	Uptake of MITS
	Only necessary if investigations and diagnosis is inconclusive
	Readiness of healthcare providers for performing the MITS procedure
	Logistical issues influencing acceptability of MITS procedure
Perceived benefits of MITS procedure	Greater diagnostic accuracy
	Identifying less common causes
Facilitators for the implementation of MITS	Building trust
	Window of opportunity
	Effective counseling is the key
	Accelerate turnaround times
Health system requirements for implementing MITS procedure	Acceptance and governance
	Equipped healthcare facilities
	Skills and training
	Cost implications

### Acceptability of MITS

#### Uptake of MITS

Public health experts acknowledged that the availability of a less-invasive autopsy procedure at the health facility could increase the willingness for cause of death assessments by parents. Moreover, health professionals in all FGDs suggested that an increase of MITS is likely in cases where parents have experienced multiple neonatal deaths, stillbirths or miscarriages. However, one neonatologist mentioned that some parents would have concerns as the results may highlight a maternal cause for which mother would have consequences from her family.

*“For a mother, there’s a concern that if she would agree for MITS procedure for her deceased baby and something unanticipated comes out, like maternal infection or a genetic reason, then her in-laws and husband will coerce her, because the death occurred due to maternal cause” (Neonatologist, KII)*

In addition, a few health professionals felt that the state of mind of family members around the time of death would affect the acceptability of MITS. Nurses mentioned that it would be challenging to approach parents who had recently lost their child as they would be experiencing grief.

#### Only necessary if investigations and diagnosis is inconclusive

Healthcare providers believed that MITS involved an advanced approach and should only be used, when the pre-death investigations are inconclusive. A few doctors showed reluctance to have MITS performed in cases where the CoD is clear such as congenital malformations, low birth weight, or birth asphyxia. Some health professionals also argued that MITS is unnecessary as there is already sufficient evidence available on the causes of stillbirths and neonatal deaths. In cases where the CoD is not obvious, health professionals suggested that the MITS procedure be carried out by a trained expert. However, a central concern related to whether one could reach the definite cause of death with MITS as the tests would be performed on dead tissues.

*“What if we do this procedure and nothing novel is discovered? What would we say? There is a lot of uncertainty in this, because it is something new, and we don’t know whether it will add any value to the existing understanding of CoD.” (Gynecologist, KII)*

#### Readiness of healthcare providers for performing the MITS procedure

Bioethics experts emphasized that it is important to know the readiness of professionals towards performing the MITS procedure. Experts believe that health professionals’ should not be trained on MITS if they are reluctant because it is unethical to force professionals’ to go against their belief and values.

*“Healthcare providers should first need to explore whether or not they would be willing to learn and perform MITS technique to rule out the CoD in neonates and stillbirths. If health professionals are performing the procedure because they are being forced by the management or supervisor, then the provider should not do it.” (Bioethics expert, KII)*

#### Logistical challenges influencing acceptability of MITS

Healthcare providers identified a few logistical challenges that could affect the acceptance and implementation of MITS. The lack of mortuary services was considered to be a major barrier since there is no separate place to store the body until the MITS procedure is conducted.

*“We do not have separate space to keep the dead bodies until the MITS procedure room is prepared.” (Health care professional, FGD)*

A few healthcare providers mentioned that families from distant places would not allow the procedure since they would like to go back to their villages soon after the death to carry out the rituals. Health professionals further elaborated that in cases where parents would show willingness for the procedure, they may require transport back to their villages.

*“Often people have to go back to their villages, they require transport facility. So if you are taking the consent then you need to be very sure that these technical things get fulfilled with utter respect.” (Health care provider, FGD)*

### Perceived benefits of MITS procedure

#### Greater diagnostic accuracy

Generally, most healthcare providers and key-informants were positive about the concept of MITS and showed willingness to adopt this technique at their health facility as it might offer greater diagnostic accuracy. Health professionals mentioned that verbal autopsies have been the most common yet inaccurate method for investigating the CoD. Experts further highlighted that MITS has the potential to correctly diagnose the causes of death as it involves body imaging and needle biopsies of organs for histopathologic and microbiologic examination. The biopsy and PCR techniques involved in this procedure were thought to be valuable for determining the specific organism that caused neonatal death or stillbirth.

*“We generally don’t know the organism that has led to the death of the child. We are hoping that once we are doing the biopsy and PCR, we’ll also know the organism that is involved in that. And once you know the organism, then perhaps their virulence and their subtypes would lead to the development of even newer vaccines.” [Neonatologist, KII]*

#### Identifying less common causes

Healthcare providers considered MITS as an important contribution to science because it has a potential to identify the less common causes of neonatal deaths and stillbirths. The procedure was considered unique as it may provide valuable insights about disease epidemiology and related treatments, which will eventually help in saving lives of newborns. One key-informant mentioned that for many years, sepsis has been considered as the major cause of child death. The procedure will greatly contribute by revealing hidden causes and syndromes that are not diagnosed through routine investigations and assessment. The neonatologist further explained that this procedure will help improve medical knowledge and public health programs.

*“Obviously, if our assumptions of those major complications are not true, this study would help us focus on other unknown and less common causes. From years, we have been dragging “sepsis” as a major cause of death. If we will have the knowledge of other causes, we will then work on addressing those.” (Healthcare professional, FGD)*

### Factors facilitating the implementation of MITS

#### Building trust

Most health professionals mentioned that building a trusting relationship with the family members and parents of the deceased fetus or newborn is the key strategy for facilitating the implementation of MITS. To build parents’ trust, healthcare providers including doctors and nurses believed that parents would like to see their child during the procedure and therefore they suggested that parents should be allowed in the closed observation/ viewing room that overlooks the MITS procedure room. One of the most important recommendations made by study participants included making counsellors part of the attending physician’s team so that counsellors are accepted by parents and can approach them for MITS consent. In addition, it was advised that counsellors should interact with parents from the beginning so that they can build a good bond with the parents, similar to the bond often developed by the attending physician.

*“Counselors should be buddied with the attending physician’s team so that counselor can develop a trust relationship with the parents as a physician does. Plus, there is need to hire separate counselors who could work 24X7 round the clock to strengthen the bonding of counselor with the parents.” (Health care professional, FGD)*

Public health experts mentioned that to build trust with the public, the MITS procedure should be conducted by trained personnel and should not be taken for granted due to the fact that it is performed in a government hospital. In addition, it was recommended that healthcare providers provide complete and accurate information concerning the MITS procedures to the parents to avoid any misinterpretation.

#### Window time

The majority of health professionals highlighted that there would be a limited time window for seeking consent for MITS. Therefore, it would be critically important to approach parents at the right time. To facilitate the implementation of MITS, nurses suggested that parents should be approached after one hour (of death), because families experience acute grief in the first hour. Nurses further explained that families should be approached for MITS consent between two to four hours (of death), because at that time families would be relatively comfortable in making decisions about whether or not to allow the procedure. Some health professionals mentioned that a few families remain in the denial phase for a few hours and therefore it would be very challenging to approach them for MITS consent.

#### Effective counseling is the key

Healthcare providers and public health experts both emphasized the need for an effective counseling approach to facilitate the implementation of MITS. Most participants suggested that counseling should be done by a person trained for using techniques such as rapport building, active listening, respect, attention and reflection.

*“A person specialized in counseling should do it. If any random person would do it then it won’t work. If someone from the staff or doctor would do it, it would not be beneficial.” (Health care professional, FGD)*

In contrast, some health professionals recommended that counseling should be done by the primary attending physician, as parents and families have established a strong trusting relationship with the child’s physician.

*“Primary physicians should initiate the counseling because if I am meeting my doctor on a daily basis, I have developed trust on him. I have a belief that whatever he is saying is right as he knows my child’s case from the beginning.” (Health care professional, FGD)*

In addition, bioethics experts indicated that the counselor should remain neutral and avoid making assumptions or unduly influencing others. Nurses highlighted that religious leaders should be part of counseling team as most parents would want to know the religious law and rulings pertaining to the MITS procedure.

#### Accelerate procedure times

Key-informants highlighted the significance of the quick procedure times and suggested that facilities and healthcare providers should be prepared and be able to complete the procedure within a few hours so that the body could be released for burial. Additionally, healthcare providers mentioned that short procedure times would potentially increase the acceptability for the MITS procedure.

*“Procedure should be done within a few hours and the facilities should be there to, for the procedure to be done quickly and efficiently and handover the bodies to the parent.” [Neonatologist, KII]*

### Health care system requirements for implementing MITS procedure

#### Acceptance and governance

One neonatologist suggested that in order to increase acceptance of MITS, it is important to have buy-in from all relevant stakeholders including government stakeholders, policy makers, implementers, researchers, religious leaders, civil society members and parents. In addition, political will and good governance were highlighted as most important factors contributing to the acceptance of MITS, as they would support provision of funds for staff hiring, training, and equipment.

*“I mean ultimately, there is a dependency on the government as far as the health is concerned, unless the government takes the ownership of any procedure, any treatment, any strategy, the impact is not going to be there in the long term and on a large scale. So of course the government has to take ownership of that. It is our duty to, first of all do this study and then perhaps once we are convinced, then pass over the information to the government that such procedure is beneficial for the community, should be adopted, necessary management should be made, have procedures like this available.” (Neonatologist, KII)*

#### Equipped healthcare facilities

Public health experts acknowledged that successful implementation of MITS would require health care facilities to be well-equipped, including both the availability of equipment and trained healthcare providers. Other key challenges to the successful implementation of MITS related to logistics, including shortage of human resources, lack of trained health professionals, inadequate funds for procuring MITS equipment, unavailability of MRI and CT machines and the lack of infrastructure.

*“We have very little man power and there is always a shortage of staff for routine care. For implementation of this new technique, we cannot overburden them.” (Health care provider in an FGD)*

#### Skills and training

One of the most frequent concerns around MITS implementation included the need to train counsellors, technicians, radiologists and pathologists to enable them to set up and sustain the service. Others reported that adequate training health professionals is essential to ensure that providers have sufficient understanding of the counseling techniques. Further, experts suggested that a multidisciplinary approach would be useful to ensure that all professionals including pathologists, radiologists, technicians, implementation managers and healthcare providers are working together for the successful implementation of MITS.

#### Cost implications

Healthcare providers argued that there are high costs associated with the implementation of MITS. Providers further explained that high costs would be a limiting factor as it would cause additional anxiety among parents of the deceased. On the other hand, a few health professionals confirmed that costs would not be a major concern if there was a buy-in from the government. Public health experts mentioned that the initial investments may be higher for setting up the infrastructure and procuring required equipment and technology; however, the operating costs may not be very high.

*“If it’s a minimal invasive tissue sampling, then of course cost is not going to be a major problem or a limiting factor. Of course, the initial investment would be high but the operating costs would not be that much.” (Neonatologist, KII)*

## Discussion

This formative research provided a unique opportunity to explore health professionals’ views and attitudes towards MITS. Such insights are crucial to ensure successful implementation and integration of new techniques within the existing health system. The study highlighted that the greatest uptake for MITS is anticipated among parents who have experienced multiple neonatal deaths, stillbirths or miscarriages. Similar to our study, a previous study conducted by Ben-sasi et al. also recognized that availability of a less-invasive autopsy procedure at the health facility would itself increase the uptake and acceptability of MITS by parents [16].

The study made an attempt to identify the factors that might influence the acceptability of MITS among health professionals in Pakistan. Most of the findings of health professionals’ perceptions of MITS are consistent with other studies [13]. Generally, MITS was considered as a positive development for the health system, and an appropriate alternative to full-autopsy. However, a few health professionals suggested that MITS should only be conducted when pre-death investigations and diagnoses are inconclusive. This highlights the importance of further research to understand and determine the criteria needed to conduct MITS. As in prior studies, this study noted that much of the success of the procedure adoption is highly dependent on health professionals’ perceptions of MITS; thus it is critical to explore providers’ comfort level with the MITS procedure [13]. Evidence also indicates that the lack of consensus by providers for new strategies relates to the lack of current knowledge about potentially effective interventions [17]. Therefore, in order to improve the acceptance of new innovations in the clinical practice, it is import to create awareness among clinicians about recent guidelines and strategies.

Greater diagnostic accuracy and identification of less common causes were identified as two main benefits of MITS by health professionals’. This is consistent with the findings of Castillo et al. suggesting that MITS is a feasible and reliable tool to improve the knowledge of CoD in developing countries [18]. In addition to these benefits, previous studies have reported that MITS procedure will eventually contribute to increasing autopsy rates, improving medical feedback to clinicians, and better overall health care quality [19].

The challenges associated with obtaining informed consent for post-mortem procedures from bereaved parents shortly after the death of their child have been reported in a number of studies [20–23]. To address these challenges, this study highlighted a number of facilitators for acceptability of MITS such as effective counselling, building trust with parents, fast-turnaround times, and approaching families between two to four hours of death in consideration of the needs for a quick burial. The study suggested that to ensure effective counselling, it is critical to train counselors on effective counseling skills and involve them in the physician’s team prior to the death of the child. As with previous studies [20, 22], this study also found that being introduced to MITS by a primary attending physician who explains the benefits of and addresses the concerns about MITS could also be a facilitator for acceptability of MITS. This indicates that involving attending physicians in the consenting process may increase the consent rate for MITS when a relationship of trust has been established between physician and parents. The recommended strategies, while realistic, demand specialized trainings on counselling and support from clinicians, hospital staff, and management as well as other hospital decision makers.

The practical challenges identified in this research when considering MITS implementation in existing healthcare systems include, lack of buy-in from government stakeholders and policy makers, lack of trained and skilled staff, poorly equipped healthcare facilities and high cost associated with the implementation of MITS. This highlights the need of engaging key stakeholders from the very beginning of the MITS implementation program to ensure that the network of main stakeholders becomes major supporters of this implementation, rather than its principal opponent.

An important limitation of this study is that the results represent a specific group of health professionals’ working in the Sindh province of Pakistan; and thus the opinions of health professionals outside Pakistan may be different. Also, the limited knowledge of MITS among healthcare professionals might have biased study findings and influenced study validity. Moreover, MITS acceptability among health professionals was explored under hypothetical conditions, as MITS had not been implemented yet. Therefore, there is a need to validate these findings in real-life setting where MITS will be implemented. Future research is required to understand the potential barriers and facilitators of implementing MITS in tertiary healthcare settings of Pakistan.

## Conclusion

In general, MITS was considered as a positive development for the health facility, health system, and particularly for communities where full-autopsy is considered as culturally and religiously unacceptable. Findings from this research are essential in understanding challenges associated with the implementation of MITS in the context of Pakistan. The facilitating factors recommended by health professionals would help to craft appropriate strategies to ensure successful implementation and integration of MITS into the existing healthcare system.

## Data Availability

The datasets used and/or analysed during the current study are available from the corresponding author on reasonable request.

## Appendix

### Semi-Structured Interview Guide

1. **Pregnancy and Birth (perceptions)**
  1.1 In your opinion what helps a woman to be healthy during her pregnancy?
    *Probes:*

- Nutritional Practices
- Antenatal visits
  1.2 In your opinion what are the causes (pregnancy-related) which result in premature birth or a stillbirth?
    *Probes:*
- Common beliefs and practices around early pregnancy loss, stillbirth, or neonatal death?
  1.3 What are the barriers to seeking care?
    *Probes:*
- Financial limitations
- Poor access to health facilities

2. **Neonate Death/Stillbirth and related practices**
  2.1 Please describe what happens when a premature or mature baby (stillbirth/ neonatal death) dies
    *Probes:*

- Chronology of events
- Parents/families interacting with the body
- Burial and mourning Process
- Cultural practices and rituals – different ethnic and religious groups. Why are those things (cultural practices) done? What happens if they’re not done?
- Cultural and religious beliefs around death

3. **Cause of Child Death**
  3.1 Do you think it is important to inquire the cause of child death?
    Probes:

- If yes why? If no why?
- How the cause of death can be determined? Do you know about any such procedure?
  3.2 To find out the cause of child death (still birth/ neonatal detah), various lab tests and samples (fluids) from the body (tissues) are taken within 24 h after a child dies. Do you thing such procedures are important?
    *Probes:*
- Do you think finding out this information would be valuable?
- If it’s valuable, why? If not, why not?
- How much or what information would be valued?
  3.3 In your opinion, would it be acceptable to perform MITS procedure to the recently deceased child?
    *Probes:*
- If yes why? If no why?

4. **Perceived advantages, facilitators and barriers related for the implementation of minimal invasive tissue sampling procedure**
  4.1 What are the perceived (foreseen) advantages for the implementation of MITS procedure?
    *Probes:*

- To understand the cause of death in stillbirth/deceased neonate
- To prevent further deaths
- Greater diagnostic accuracy
- Involves tissue analysis (to identify if it’s an infection)
- Comparatively shorter procedure (accelerate turnaround times)
- Procedure more palatable (pleasant)
  4.2 What are the concerns for the use of MITS procedure in a deceased neonate/stillbirth?
    *Probes:*
- Concerns related to body/soul
- Concerns with timing of ceremonies and burial
- Religious beliefs
- Traditional beliefs
- Fear of breach of confidentiality (in relation to the disease carrying stigma e.g. HIV)
- Perceived inappropriateness (in cases when clinical diagnosis is clear)
- Not reaching same level of certainty
- Complex decision making process
- MITS procedure costs for the family
- State of mind around the death
  4.3 What are the perceived facilitators for the implementation of MITS procedure?
    *Probes:*
- Carrying out the procedure ASAP to facilitate timely body release, burial and related ceremonies
- Body preservation
- Community involvement (support from leaders, health professionals)
- Information and transparency (clear information about the procedure)
- Cost reduction (waiving the cost of MITS procedure)

5. **Suggestions to improve awareness about MITS procedure**
  5.1 What do you think would be the best method of educating the community about MITS?
    *Probes:*

- Community discussions
- Counseling of parents/families

6. **Requirements for the health system for MITS procedure** (Questions only for health system and public health experts)
  6.1 What are some of the requirements for the health system (i.e. medical facilities) to conduct MITS procedures?
    *Probes:*

- Level of current knowledge (about MITS) among health care workers.
- Acceptability of MITS among health care workers.
- Availability of experts to conduct MITS/personnel
- Equipment
- Healthcare facilities – good reputation of the facilities performing MITS
- Health professionals attitude and preparedness
- Integration of MITS within the existing health system
  6.2 Having named those requirements, which of them are in place in your health system?
    *Probes:*
- What would need to be put in place in regard to facilities? Equipment? Personnel?
- Is the health system prepared?
- Unprepared health system (lack of equipment, financial limitations)
  6.3 What role could your health system play in carrying out MITS?
    *Probes:*
- Could MITS be carried out in your health facilities?
- Could your healthcare workers go out into the community to carry out MITS?
  6.4 What are the perceived implementation issues relating to the MITS procedure?
    *Probes:*
- Lack of skills and training
- Logistics
- Cost implications
- Equity concerns – access
- Acceptance and governance
- Reluctance from healthcare professionals (increased workload)

7. **Role of government (questions only for government authorities)**
  7.1 What is the role of the government, if any, when a child dies?
    *Probes:*

- What are the reporting requirements?
- Are there any investigations conducted (i.e. if there is suspicion of intentional injury causing the death)?
  7.2 What government stakeholders think about MITS procedure?
    *Probes:*
- Is it acceptable and feasible?
- Can be supported by government?

## Abbreviations

CDA: Complete Diagnostic Autopsy
CoD: Cause of Death
ERC: Ethical Review Committee
FGDs: Focus Group Discussions
KIIs: Key-informant Interviews
MITS: Minimal Invasive Tissue Sampling
NICH: National Institute of Child Health
PURPOSe: Project to Understand and Research Preterm Pregnancy Outcome in South Asia
